# Effect of Edaravone Combined with Anticoagulant Therapy on the Serum hs-CRP, IL-6, and TNF-*α* Levels and Activity of Daily Living in Patients with Acute Cerebral Infarction

**DOI:** 10.1155/2022/8603146

**Published:** 2022-02-28

**Authors:** Chao Sun, Cuiling Ma, Yu Sun, Lili Ma

**Affiliations:** ^1^Department of Neurology, Yantaishan Hospital, Yantai 264000, Shandong, China; ^2^Department of Neurology, The People's Hospital of Feicheng, Feicheng 271600, Shandong, China

## Abstract

**Objective:**

To explore the effect of edaravone combined with anticoagulant therapy on the serum hs-CRP, IL-6, and TNF-*α* levels and the activity of daily living (ADL) in patients with acute cerebral infarction (ACI).

**Methods:**

The clinical data of 84 ACI patients treated in our hospital from August 2020 to August 2021 were retrospectively analyzed, and they were divided into the routine group (*n* = 42) and the combined group (*n* = 42) according to the order of admission. Both groups were treated with routine clinical treatment, and the combined group was additionally treated with edaravone combined with anticoagulant therapy. Serum samples were collected from both groups after treatment. ELISA was used to detect the serum inflammatory factor levels, and the modified Barthel index score was used to evaluate the ADL of patients.

**Results:**

Compared with the routine group, the combined group achieved obviously lower levels of PMA, CD62p, and serum inflammatory factors after treatment (*P* < 0.001), higher modified Barthel score after treatment (*P* < 0.001), lower plasma viscosity, platelet aggregation rate, and plasma fibrinogen level after treatment (*P* < 0.001), and higher clinical overall efficacy (*P* < 0.05).

**Conclusion:**

Edaravone combined with anticoagulant therapy is a reliable method to enhance ADL and reduce the inflammatory response of ACI patients. This strategy greatly reduces the platelet-activating factor levels of patients and improves the comprehensive clinical efficacy, and its further research will help to establish a better solution for these patients.

## 1. Introduction

Acute cerebral infarction (ACI) refers to brain tissue necrosis caused by the sudden interruption of cerebral blood supply, with complicated pathogenesis [1]. Its etiology may be related to cerebral artery stenosis and blockage caused by abnormal blood vessels, blood, and hemodynamics [2]. With acute onset, rapid progression, and the clinical manifestations of most patients as tinnitus, headache, slurred speech, and vomiting, this disease damages the neurological function and leads to a poor prognosis. With the aggravation of aging and lifestyle changes in China, the clinical incidence of ACI has been rising by year and developing toward a younger age, and its clinical diagnosis and treatment have become the focus of social concern [3]. A large number of clinical studies [4, 5] have confirmed that effective dredging of infarction lesions and improvement of neurological function at an early stage are the key factors affecting the prognosis of patients. At present, antiplatelet drugs such as aspirin, ozagrel, and clopidogrel are mostly used in clinic, but the efficacy remains unsatisfactory [6]. Edaravone, a free radical scavenger, can improve the local blood flow of cerebral infarction lesions, prevent the disease progression, and alleviate neurological symptoms, with confirmed efficacy in diseases such as acute carbon monoxide poisoning, cardiogenic cerebral infarction, and hypertensive cerebral hemorrhage [7–9]. Although not recommended in the guidelines, anticoagulant therapy for ACI is very common in foreign countries, with the common anticoagulant drugs such as aspirin, warfarin, and plavix. From the perspective of pathophysiological mechanism, anticoagulant therapy can restrain the deterioration of neurological symptoms, prevent the recurrence of early stroke, and improve microcirculation and blood supply [10]. However, the current research on anticoagulant therapy for ACI is still in the initial stage, lacking sufficient evidence-based proof [11]. At present, few studies have reported the efficacy of edaravone combined with anticoagulant therapy on ACI. Based on this, the ACI patients admitted to our hospital were retrospectively analyzed and received different treatment regimens after admission, aiming to observe whether edaravone combined with anticoagulant therapy can benefit ACI patients in terms of clinical effect, reported as follows.

## 2. Materials and Methods

### 2.1. Clinical Data

The clinical data of 84 ACI patients treated in our hospital from August 2020 to August 2021 were retrospectively analyzed, and they were divided into the routine group (*n* = 42) and the combined group (*n* = 42) according to the order of admission. This study was in line with the Declaration of Helsinki (as revised in 2013) [12].

  Inclusion criteria are as follows: (1) the enrolled subjects all met the diagnostic criteria of ACI in Chinese Guidelines for Diagnosis and Treatment of Acute Ischemic Stroke (2010) [13], and the infarction lesions were confirmed by MRI or CT scan, with the CT images showing low-density lesions and the symptoms such as tinnitus, vertigo, nausea, vomiting, and coma; (2) all patients were treated within 72 hours after onset, and had the first onset; and (3) patients had no allergic history for the drugs used in this treatment, with clear consciousness.
  Exclusion criteria are as follows: (1) the patients with serious injury of other vital organs; (2) patients complicated with coagulation disorders; (3) patients who had received anticoagulant treatment before; and (4) patients who had the diseases with hemorrhagic tendency.

### 2.2. Treatment Methods

Both groups received routine treatment after hospitalization, including basic treatments such as lowering intracranial pressure, regulating water-electrolyte imbalance, improving microcirculation, antihypertension, and oxygen inhalation.

The combined group was additionally treated with edaravone combined with anticoagulant therapy. 30 mg of edaravone (manufacturer: China National Medicines Guorui Pharmaceutical Co., Ltd.; NMPA approval no.: H20080056; specification: 20 ml/30 mg) was dissolved in 100 ml of isotonic saline and then was intravenously dripped into the patients for continuous treatment of 14 days, twice a day. At the same time, anticoagulant therapy was performed through the subcutaneous injection of 5000 IU of low molecular weight heparin calcium (manufacturer: Hebei Changshan Biochemical Pharmaceutical Co., Ltd.; NMPA approval no.: H20063909; specification: 0.2 ml: 2050AXaIUx2 vials/box) for continuous treatment of 14 days, once every 12 hours.

### 2.3. Observation Indexes

Fasting elbow venous blood (5 mL) was collected in the morning from both groups after treatment and centrifuged at 3000 *r*/min for 15 min. The serum was taken and stored in a refrigerator at −80°C for detection. The XTG-1600E flow cytometry (manufacturer: Shanghai Huanxi Medical Device Co., Ltd.) was used to detect the serum platelet-activating factors, including the levels of platelet-monocyte aggregation (PMA) and *α*-granulosa glycoprotein (CD62p). ELISA was adopted to detect the serum inflammatory factor levels, including interleukin-6 (IL-6), high-sensitivity C-reactive protein (hs-CRP), and tumor necrosis factor-*α* (TNF-*α*). The kits were purchased from Shenzhen Xinbosheng Biological Co., Ltd., and the detection was performed strictly in accordance with the kit instructions.

Hemorheology indexes: 4 ml of peripheral venous blood was collected after treatment, and a hemorheological analyzer (manufacturer: Dongguan Maiyue Medical Device Co., Ltd.; model: HL-5000) was used to detect the plasma fibrinogen, platelet aggregation rate, and plasma viscosity.

The modified Barthel Index Scale [14] was used to evaluate the activity of daily living (ADL) of patients, including 11 items such as diet, bathing, dressing, and walking. Each activity was rated in five levels, and different levels represented different levels of independent ability. The lowest level was level 1, and the highest level was level 5, and a higher level indicated higher independent ability. The patients with a score ≥60 points could basically take care of themselves; those with 41–59 had moderate dysfunction and needed help from others in daily life; those with 21–40 had severe dysfunction, with obviously life dependence; and those with a score ≤20 were completely dependent on others. The specific scoring criteria are shown in Table 1.

Evaluation of overall efficacy after treatment: the European Stroke Scale (ESS) [15] was used to evaluate the clinical efficacy of patients before and after treatment. The scale had 14 items, including consciousness level, language, visual field, finger muscle strength, and gait, with a total score of 100 points. A higher score represented a better function of the subjects.

If the ESS score increased by 85%–100%, the patients were cured; if the ESS score increased by 50%–84%, the treatment was markedly effective; if the ESS score increased by 20%–49%, the treatment was effective; and if the ESS score increased by less than 20%, the treatment was ineffective. Total effective rate = (cured cases + markedly effective cases)/total cases × 100%.

### 2.4. Statistical Methods

The data in the study were processed by the professional statistical software SPSS23.0 and graphed by GraphPad Prism 7 (GraphPad Software, San Diego, USA). The enumeration data were tested by *χ*^2^ and expressed as *n*(%), while the measurement data were tested by the *t* test and expressed as mean ± SD. When *P* < 0.05, the differences were statistically significant.

## 3. Results

### 3.1. Comparison of Clinical Data

No notable differences in clinical data such as gender ratio, onset time, diseased sites, and disease types were observed between the two groups (*P* > 0.05), see Table 2.

### 3.2. Comparison of Platelet-Activating Factors

After treatment, the PMA and CD62p levels in the combined group were obviously lower compared with the routine group (*P* < 0.001), see Figure 1.

### 3.3. Comparison of Serum Inflammatory Factor Levels

After treatment, the various serum inflammatory factor levels were obviously lower in the combined group than in the routine group (*P* < 0.001), see Table 3.

### 3.4. Comparison of Hemorheology Indexes

After treatment, plasma viscosity, platelet aggregation rate, and plasma fibrinogen level in the combined group were remarkably lower compared with the routine group (*P* < 0.001), see Table 4.

### 3.5. Comparison of Modified Barthel Scores

The modified Barthel score in the combined group after treatment was obviously higher compared with the routine group (*P* < 0.001), see Figure 2.

### 3.6. Comparison of Overall Efficacy after Treatment

The total clinical effective rate of the combined group was markedly higher than the routine group (*P* < 0.05), see Table 5.

## 4. Discussion

Relevant epidemiological investigation [16] shows that ACI has become the second leading cause of death worldwide. As a common and frequently-occurring disease in clinic, ACI is characterized by high morbidity, mortality, disability, and recurrence. The abnormal blood supply of local brain tissues caused by various factors leads to brain tissue lesions and damages the brain tissues, triggering ACI. With acute onset and rapid progression, ACI patients have a poor prognosis and are prone to sequelae such as hemiplegia, hemiparesis, and language barriers, seriously affecting their physical and mental health and quality of life [17]. At present, ACI is mainly treated with anticoagulation, thrombolysis, and lipid-lowering to stabilize plaques. The common side effect of thrombolytic therapy is bleeding, which can manifest as skin and mucosa bleeding in patients with mild symptoms and visceral hemorrhage, such as gastrointestinal bleeding and brain bleeding, in patients with severe symptoms. Lipid-lowering drugs to stabilize plaque drugs often lead to gastrointestinal adverse reactions, such as upper abdominal discomfort and nausea as well as muscle weakness or pain, in a small number of patients. A study [18] has found that fibrinogen increases and the body is in a hypercoagulable state in ACI patients because the impaired vascular endothelium triggers large consumption of anticoagulant factors such as antithrombin III (AT3) in the fibrinolytic process, promoting the formation of the hypercoagulable state to a certain extent. Due to the hypercoagulable state, low anticoagulant state, and fibrinolytic dysfunction, the reduced blood perfusion in the ischemic area, poor collateral circulation compensation, and expansion of thrombosis will result in the disease progression [19], suggesting that anticoagulant therapy should be given in time after the onset of ACI. However, conventional anticoagulant therapy may increase the risk of bleeding complications. Therefore, it is still controversial about anticoagulant therapy for acute ACI.

A clinical study [20] has shown that the short-term application of low molecular weight heparin in mild ACI is safe and effective. The effect of the anticoagulant factor Xa of low molecular weight heparin is 2–4 times that of unfractionated heparin, while the anticoagulant factor IIa has a weak effect, so the incidence of bleeding risk is significantly lower than that of unfractionated heparin. A domestic clinical control trial [21] showed that after patients in the control group orally took 100 mg of aspirin once a day, while the observation group additionally received the subcutaneous injection of low molecular weight heparin (5000 IU), twice a day, the National Institutes of Health Stroke Scale (NIHSS) score and cerebral infarction improvement in the observation group after treatment were better than those in the control group (*P* < 0.05), which confirmed the better effect of anticoagulant therapy. While removing the free radicals in the injured parts, edaravone, a neuroprotective agent, can reduce the damage and apoptosis of nerve cells, improve the survival of nerve cells in the ischemic parts of the brain and reduce the damaged area of cerebral infarction, thus promoting the recovery of blood supply for injured brain tissues [22].

Hypoxia, ischemia, and blood supply disorders in local brain tissues can activate microglia and peripheral white blood cells, resulting in a series of inflammatory reactions in the body and aggravating the damage of brain tissues and peripheral neurons. A previous study [23] has shown that inflammatory factors such as IL-6, IL-8, and hs-CRP can promote the formation of thrombosis, among which hs-CRP is an important indicator reflecting atherosclerosis and acute inflammatory response. In this study, after edaravone combined with anticoagulant therapy was adopted, the serum inflammatory factor levels in the combined group after treatment were notably lower than those in the routine group (*P* < 0.001), suggesting that the combined therapy can effectively alleviate the inflammatory response of ACI patients and then delay the disease progression. ACI patients have a high risk of sequelae for the special nerve cells, resulting in the decrease of ADL in patients. Therefore, effective treatment programs to improve the ADL of patients have become the key to improving the prognosis of the disease [24]. In this study, it was found that the modified Barthel score after treatment was obviously higher in ACI patients who received edaravone combined with anticoagulant therapy than in those with routine treatment, indicating that the combined therapy can reduce perfusion injury of cerebral cells and improve the ADL of patients. The study also has some shortcomings. For example, the small sample size of ACI patients indicates the possible selection bias. In addition, the adverse reactions of patients after treatment are not studied. Therefore, it is necessary to expand the sample size and conduct more multicenter studies to further confirm the results of the study.

In conclusion, edaravone combined with anticoagulant therapy is a reliable method to reduce the serum inflammatory factor levels, improve the hemorheology indexes, and enhance the ADL of ACI patients. Therefore, its further research will help to establish a better solution for such patients.

## Figures and Tables

**Figure 1:** Comparison of platelet-activating factors after treatment (mean ± SD). (a) comparison of PMA levels after treatment. The abscissa represented the routine group and combined group, and the ordinate represented the PMA level (%). The average PMA levels of the routine group and combined group after treatment were (21.42 ± 2.42) % and (17.72 ± 2.00) %. ^∗^ indicated a notable difference in the average PMA levels between the two groups after treatment (*t* = 7.638, *P* < 0.001). (b) Comparison of CD62p levels after treatment. The abscissa represented the routine group and combined group, and the ordinate represented the CD62p level (%). The average CD62p levels of the routine group and combined group after treatment were (2.56 ± 0.20) % and (1.29 ± 0.19) %. ^∗∗^ indicated a notable difference in the average CD62p levels between the two groups after treatment (*t* = 29.836, *P* < 0.001).

**Figure 2:** Comparison of modified Barthel scores after treatment (mean ± SD). The abscissa represented the routine group and combined group, and the ordinate represented the modified Barthel score (points). The modified Barthel scores of the routine group and combined group after treatment were (54.86 ± 4.96) and (65.40 ± 5.61). ^∗^indicated a notable difference in the modified Barthel scores after treatment between the two groups (*t* = 9.122, *P* < 0.001).

**Table 1:** Scoring criteria of modified Barthel Index Scale.

Assessment items	Complete dependence level 1	Maximum help level 2	Medium help level 3	Minimum help level 4	Complete independence level 5
Diet	0	2	5	8	10
Defecation	0	2	5	8	10
Bathing	0	1	3	4	5
Decoration	0	1	3	4	5
Walking	0	3	8	12	15
Stool control	0	2	5	8	10
Urine control	0	2	5	8	10
Stairs climbing	0	2	5	8	10
Movement of beds and chairs	0	3	8	12	15
Dressing	0	2	5	8	10
Sitting in a wheelchair^*∗*^	0	1	3	4	5

^∗^indicated that this item was assessed only when the patients were not able to walk.

**Table 2:** Comparison of clinical data (*n* = 42).

Items	Routine group	Combined group	*χ* ^2^/*t*	*P* value
Gender			0.192	0.661
Male/female	24/18	22/20		
Body weight (mean ± SD, kg)	73.16 ± 5.43	73.41 ± 5.90	0.202	0.840
Average age (mean ± SD, years old)	60.38 ± 3.77	60.74 ± 3.39	0.460	0.647
Onset time (mean ± SD, h)	23.45 ± 4.61	23.83 ± 3.94	0.406	0.686
*Diseased sites*				
Brainstem	15 (35.71)	13 (30.95)	0.214	0.643
Internal capsule	21 (50.00)	19 (45.24)	0.191	0.662
Lateral frontotemporal lobe	6 (14.29)	10 (23.81)	1.235	0.266
*Combined diseases*				
Hyperlipidemia	8 (19.05)	9 (21.43)	0.074	0.786
Hypertension	14 (33.33)	12 (28.57)	0.223	0.637
Coronary heart disease	15 (35.71)	13 (30.95)	0.214	0.643
Diabetes	5 (11.90)	8 (19.05)	0.819	0.365
Smoking history	13 (30.95)	16 (38.10)	0.474	0.491
Drinking history	17 (40.48)	19 (45.24)	0.194	0.659
*Disease types*				
Monofocal type	18 (42.86)	16 (38.10)	0.198	0.657
Multifocal type	10 (23.81)	13 (30.95)	0.539	0.463
Lacunar type	14 (33.33)	13 (30.95)	0.055	0.815
*Marital status*				
Married	35 (83.33)	37 (88.10)	0.389	0.533
Unmarried	4 (9.52)	3 (7.14)	0.156	0.693
Divorced	3 (7.14)	2 (4.76)	0.213	0.645
Residence			0.192	0.661
Urban area	18 (42.86)	20 (47.62)		
Rural area	24 (57.14)	22 (52.38)		

**Table 3:** Comparison of serum inflammatory factor levels after treatment (mean ± SD).

Group	*n*	hs-CRP (*μ*g/L)	IL-6 (ng/L)	TNF-*α* (ng/L)
Routine group	42	16.52 ± 1.38	62.90 ± 3.04	287.87 ± 13.31
Combined group	42	10.77 ± 1.41	48.15 ± 2.95	132.95 ± 12.78
*t*		18.888	22.566	54.411
*P* value		<0.001	<0.001	<0.001

**Table 4:** Comparison of hemorheology indexes after treatment (mean ± SD).

Group	*n*	Plasma viscosity (MPa·s)	Platelet aggregation rate (%)	Plasma fibrinogen (g/L)
Routine group	42	5.54 ± 0.59	55.44 ± 5.96	5.34 ± 0.68
Combined group	42	4.36 ± 0.65	48.17 ± 6.06	3.46 ± 0.67
*t*		8.711	5.543	12.763
*P* value		<0.001	<0.001	<0.001

**Table 5:** Comparison of overall efficacy after treatment (*n* (%)).

Group	*n*	Cured	Markedly effective	Effective	Ineffective	Total effective rate
Combined group	42	13 (30.95)	24 (57.14)	3 (7.14)	2 (4.76)	88.10% (37/42)
Routine group	42	11 (26.19)	18 (42.86)	8 (19.05)	5 (11.90)	69.05% (29/42)
*χ* ^2^						4.525
*P* value						<0.05

## Data Availability

The data used to support the findings of this study are available on reasonable request from the corresponding author.
